# MCU That Is Transcriptionally Regulated by Nrf2 Augments Malignant Biological Behaviors in Oral Squamous Cell Carcinoma Cells

This article has been retracted.

**DOI:** 10.1155/2021/6650791

**Published:** 2021-06-03

**Authors:** Ran Wu, Weiwen Zuo, Xiaoliang Xu, Lei Bi, Chunguang Zhang, Hui Chen, Hui Liu

**Affiliations:** ^1^Department of Stomatology, North China University of Science and Technology Affiliated Hospital, Tangshan, 063000 Hebei, China; ^2^Department of Stomatology, Tangshan Vocational and Technical College, Tangshan, 063000 Hebei, China; ^3^Department of Stomatology, The Second Hospital of Tangshan, Tangshan, 063000 Hebei, China

## Abstract

**Objective:**

To clarify the role and molecular mechanism of mitochondrial calcium uniporter (MCU) in the malignant biological behaviors of oral squamous cell carcinoma (OSCC) cells through clinical and cellular experiments.

**Methods:**

Immunohistochemistry and qRT-PCR techniques were used to observe the expression of MCU, nuclear factor erythroid 2-related factor 2 (Nrf2), mitochondrial calcium uptake 1 (MICU1), and MICU2 in OSCC and normal tissues. After treatment with si-MCU, spermine, and/or sh-Nrf2, malignant biological behaviors of OSCC cells including proliferation, migration, and apoptosis were detected by clone formation, migration, and mitochondrial membrane potential (MMP) assays. Furthermore, MCU, MICU1, MICU2, Nrf2, and other proteins related to malignant biological behaviors were examined using western blot, immunohistochemistry, and immunofluorescence assays.

**Results:**

MCU, Nrf2, and MICU1 were strongly expressed in OSCC as compared to normal tissues, while MICU2 was relatively weakly expressed in OSCC tissues. Knockdown of MCU distinctly weakened proliferation and migration and lowered MMP level in CAL 27 cells. Conversely, its activation reinforced migrated capacity and increased MMP level in CAL 27 cells, which was reversed after cotransfection with sh-Nrf2. After treatment with si-MCU or spermine, Nrf2 expression was not affected in CAL 27 cells. However, MCU expression was distinctly suppressed in CAL 27 cells transfected with sh-Nrf2. Furthermore, knockdown of Nrf2 significantly reversed the increase in expression of MICU1 and MICU2 induced by MCU activation in CAL 27 cells.

**Conclusion:**

MCU, as a novel oncogene of OSCC, augments malignant biological behaviors of OSCC cells, which could be transcriptionally regulated by Nrf2.

## 1. Introduction

Oral squamous cell carcinoma (OSCC) accounts for 90% oral malignancies, characterized by high aggressive and early lymph node metastasis [1–3]. According to the latest GLOBOCAN 2019 report, the number of new cases of oral cancer in 2019 is 53,000, and the death toll is 10,860 in the United States [4]. OSCC is related to poor lifestyles such as smoking, excessive drinking, and chewing betel nut [5]. The current treatment methods for OSCC are mainly surgical resection, chemotherapy, and radiotherapy [6]. Despite the fact that the treatment is constantly improving, the scope of the operation is severely restricted because the oral surgery closely contacts important tissues and organs [7]. Furthermore, most of patients have high drug resistance and cytotoxicity. Thus, the prognosis of OSCC is still very poor, with a five-year survival rate of <50% [8]. Therefore, it is of great significance for OSCC treatment to find markers with molecular diagnosis, prognosis prediction, and targeted therapy.

Mouth is the beginning of the digestive tract and communicates with the respiratory tract. A variety of risk factors can promote tumor cells to metastasize to the submental, mandibular, and neck lymph nodes, leading to the infiltrating growth of the tumor at an early stage [9]. Moreover, tumor cells damage the surrounding organs and tissues, thereby causing some facial dysfunctions (such as loose teeth, facial paralysis, restricted mouth opening, pain, and infection), which significantly reduce the patient's quality of life [10]. The maxillofacial tissue contains a large number of blood vessels and nerves, and the incidence of neck lymph node metastasis and invasion is high [11]. Its degree of malignancy is mainly related to tumor invasion and metastasis. The pathogenesis of OSCC is due to multiple genes and multiple stages, but the specific molecular mechanism is not yet clear [12].

Intracellular Ca^2+^ homeostasis is mainly responsible for mitochondria, which participates in the regulation of various key cellular functions like cell proliferation and death [13]. The flow of Ca^2+^ into mitochondria is mainly regulated by a mitochondrial calcium uniporter (MCU) complex. The MCU complex is composed of channel-forming subunits and regulatory elements, whose activity is regulated by mitochondrial calcium uptake 1 (MICU1), MICU2, and MICU3 [14]. MICU1 and MICU2 form a disulfide-linked dimer, which binds to the MCU complex. MICU2 has been shown to inhibit MCU complexes, whose overexpression reduces the uptake of mitochondrial Ca^2+^. The decrease in MICU1 expression also leads to the loss of MICU2 in the complex. The Human Protein Atlas project funded by the Knut and Alice Wallenberg Foundation is aimed at providing information on the tissue and cell distribution of 24,000 human proteins by immunohistochemistry. Based on this project [15], in most cancer tissues, MCU shows moderate to strong immunostaining. For MICU1, moderate to strong immunostaining is also detected in most malignant tissues. For MICU2, weak to moderate immunostaining is found. Growing evidence suggests that the MCU complex is closely related to various cancers such as breast cancer [16], hepatocellular carcinoma [17], and colon cancer [18]. However, no research has reported the function of MCU in OSCC. Nrf2, a basic region-leucine zipper transcription factor, mediates the protection of cells against carcinogens and oxidative damage via transcriptionally regulating detoxification enzymes and antioxidant genes [19]. Nrf2 has a dual role in carcinogenesis and progression. On the one hand, Nrf2 protects normal cells from transforming into cancer cells [20]. On the other hand, activation of Nrf2 promotes cancer cell survival and inhibits cell apoptosis [21]. It has been reported that the activation of Nrf2 induces the cancer phenotype in OSCC cells [22]. In this study, we found that MCU expression was regulated by the transcription factor Nrf2, and it could induce malignant biological behaviors of OSCC cells, which offered novel insight into the pathogenesis of OSCC.

## 2. Materials and Methods

### 2.1. Patients and Tissues

A total of 81 OSCC tissues and adjacent normal tissues were obtained in the North China University of Science and Technology Affiliated Hospital during 2014-2016. None of them did undergo radiotherapy, chemotherapy, or immunotherapy before surgery. This experiment was approved by the Ethics Committee of North China University of Science and Technology Affiliated Hospital (2014012). The research was carried out in accordance with the World Medical Association Declaration of Helsinki, and all subjects provided written informed consent [23].

### 2.2. Immunohistochemistry

After deparaffinization and hydration, the 4 *μ*m thick sections were sealed with 100 *μ*l FBS and incubated in a humidified box for 20 min. The sections were incubated with primary antibodies against HO-1 (1 : 100; Proteintech, China; 27282-1-AP), Nrf2 (1 : 100; Proteintech, China; 16396-1-AP), MCU (1 : 100; Santa Cruz, USA; sc-515930), MICU1 (1 : 100; Abcam, USA; ab190114), MICU2 (1 : 100; Abcam, USA; ab101465), VEGF (1 : 100; Abcam, USA; ab32152), TGF-*β* (1 : 100; Abcam, USA; ab215715), HIF-1*α* (1 : 100; Abcam, USA; ab51608), N-cadherin (1 : 100; Abcam, USA; ab98952), and E-cadherin (1 : 100; Abcam, USA; ab40772) overnight in a refrigerator at 4°C. The next day, the sections were taken out of the refrigerator at 4°C and reheated in the incubator at 37°C for 45 min. Each section was incubated with 50 *μ*l of biotin-labeled Universal SAP (mouse, rabbit) secondary antibody (ZSGB-BIO, China; SAP-9100) and goat enhanced polymer secondary antibody (ZSGB-BIO, China; PV-9003) at room temperature for 1 h, followed by 50 *μ*l horseradish peroxidase-labeled streptavidin working solution at 37°C for 30 min. The sections were developed with DAB staining for 5 min. The sections were counterstained with hematoxylin for 2 min and then differentiated with hydrochloric acid and alcohol. After dehydration with gradient alcohol, the sections were cleared with xylene I and II for 10 min each. Then, the sections were mounted with neutral gum, and the results were observed under a microscope.

The semiquantitative *H*-score method was used to determine the expression levels of the target proteins. The staining intensity was divided into 4 groups: 0 points for no staining, 1 point for weak staining, 2 points for moderate staining, and 3 points for strong staining. Four fields were randomly selected. The percentage of positive cells and staining intensity point were multiplied as the final score. The immunohistochemical sections were judged independently by 2 experienced pathologists.

### 2.3. Cell Culture

Human CAL 27 cells (ZQ0606; Shanghai Zhong Qiao Xin Zhou Biotechnology Co. Ltd., China) were grown on the 90% DMEM (Gibco, Invitrogen, USA) plus 10% FBS and 1% double antibody. The cells were cultured under 5% CO_2_, 37°C constant temperature, and humidity conditions.

### 2.4. Transfection

Two shRNAs targeting the Nrf2 lentiviral plasmid purchased from HAN Biotech (Table 1) and controls were inserted into the pENTR plasmid recombined with the pBLOCK-iT™ 6-DEST vector. Adenoviral particles were prepared by using the Adenoviral Expression System (Invitrogen, USA), which were purified using the Vivapure®AdenoPACKTM20RT Kit (Sartorius, Germany). CAL 27 cells were cultivated to the logarithmic growth phase, which were then inoculated in a 10 cm culture dish (1.5 × 10^6^ cells) 2 days before transfection. When the cells grew to about 80% confluence, they were incubated with plasmids for 6-8 h. 48 h after transfection, the transfection efficiency was investigated under a fluorescence microscope, which was validated using western blot. si-MCU or control was transfected into cells via Lipofectamine 2000 (Table 1).

### 2.5. Western Blot

Tissues or cells were lysed with cell lysis buffer (Beyotime, Shanghai, China) for 20 min and then placed on ice for 20 min. The lysate was transferred onto a centrifuge tube and was centrifuged at 12000 rpm for 9 min. An appropriate amount of the supernatant was harvested and placed in a new 1.5 ml centrifuge tube at -80°C. The BCA method was utilized to determine the protein content and concentration. After the gel separation, the sample was transferred to the PVDF membrane (Millipore, USA). The membrane was blocked by the blocking solution for 30 min. Then, the membrane was incubated with primary antibodies against HO-1 (1 : 1000; Proteintech, China; 27282-1-AP), Nrf2 (1 : 1000; Proteintech, China; 16396-1-AP), MCU (1 : 1000; Santa Cruz, USA; sc-515930), MICU1 (1 : 1000; Abcam, USA; ab190114), MICU2 (1 : 1000; Abcam, USA; ab101465), vimentin (1 : 2000; Abcam, USA; ab92547), N-cadherin (1 : 1000; Abcam, USA; ab98952) and E-cadherin (1 : 2000; Abcam, USA; ab40772), and *β*-actin (1 : 1000; Proteintech, China; 20536-1-AP) overnight at 4°C. After 24 h, 5 ml TBST was added and rinsed 4 times for 5 min each time. The membrane was incubated with secondary antibodies (1 : 5000; ZSGB-BIO, China; ZB-2306, ZB-2301, and ZB-5305) at 37°C for 2 h. Following washing, ECL was used for dyeing. The optical density value of the band was analyzed utilizing the ImageJ software, which was compared with the value of the *β*-actin (internal reference) band.

### 2.6. Clone Formation Assay

The transfected cells were seeded in a 6-well plate (5 × 10^3^) and cultured in a cell incubator for about 2 weeks, during which the medium was changed every 3 days. After removing the original culture medium, the cells were stained with Giemsa working solution (500 *μ*l/well) at room temperature for 15 min. The results were observed under a microscope. The cells were counted under random 3 fields of view. The clone formation rate = the number of clones/the total number of inoculated cells × 100%.

### 2.7. Wound Healing Assay

The cells were spread into a 6-well plate (5 × 10^5^ cells/well), which were placed in a medium plus 10% FBS, and incubated in a 37°C, 5% CO_2_ incubator. After the cells adhered to the wall, they were replaced with FBS-free medium, which were then cultured overnight. Using a sterile 100 *μ*l pipette tip, the scratch experiment was performed. The original cell culture medium was discarded, and the cells were washed with PBS solution for 3 times to wash away the floating cells scraped off by scratches. Serum-free medium was added to continue the culture. The cell culture plates were taken under an inverted microscope at 0 h and 24 h and analyzed using Image-Pro Plus software. Three scratch fields were randomly selected to measure the scratch distance in each group.

### 2.8. Transwell Assay

1 × 10^5^ cells were seeded to the transwell chamber. 600 *μ*l of culture medium containing 10% FBS was added to the lower chamber of the 24-well plate and incubated for 24 h. The transwell chamber was taken out and transferred to 95% methanol for fixation for 30 min. Then, it was stained using 0.1% crystal violet staining solution for 20 min. The nonmigrated cells in the upper layer of the chamber were gently wiped off with a cotton swab. The transwell chamber was moved to a glass slide and covered with neutral gum. Under the microscope, 5 different fields of view were selected and the number of cells passing through the membrane was calculated.

### 2.9. Mitochondrial Membrane Potential

The cells were seeded in a 24-well plate (2 × 10^6^/well) and cultured routinely for 24 h to adhere to the wall. The cells were incubated with 5 *μ*g/ml JC-1 working solution in a fresh medium at 37°C for 20 min in the dark. Then, the culture medium was aspirated and the excess JC-1 dye was washed off. An appropriate amount of fresh culture medium was added to the cells. The images were observed under a fluorescence microscope. The cell membrane potential of the normal group was used as a control.

### 2.10. Immunofluorescence

Paraffin-embedded tissue sections were incubated with primary antibodies labeled with fluorescent substance against MCU (1 : 100; sc-515930; Santa Cruz, US), MICU1 (1 : 1000; Abcam, USA; ab190114), MICU2 (1 : 1000; Abcam, USA; ab101465), and Nrf2 (1 : 1000; Proteintech, China; 16396-1-AP) overnight at 4°C, followed by secondary antibodies Alexa Fluor® 488 conjugate (1/100; ZSGB-BIO, China; ZF-0311, 1/100; ZSGB-BIO, China; ZF-0514) and Alexa Fluor® 594 conjugate (#ZF-0513, 1 : 100, ZSGB-BIO, China) at room temperature for 2 h. The images were observed under an immunofluorescence microscope.

### 2.11. Cellular Immunofluorescence

Trypsinized CAL 27 cells were seeded in a 24-well plate (1 × 10^5^). When the cell fusion exceeded 50%, the cells were transfected. The cells were fixed with 4% polyformic acid for 15 min at room temperature. The cell-climbing slide was washed with 0.5% Triton X-100-containing PBS solution. After the cells were blocked with 3% BSA, they were incubated with primary antibodies against MCU, MICU1, MICU2, and Nrf2 overnight in a refrigerator at 4°C. On the second day, the cells were incubated with the secondary antibody in the dark at room temperature for 2 h, followed by DAPI solution at room temperature for 10 min. The antifluorescence quencher was dropped on the glass slide. The images were investigated with a laser scanning confocal microscope.

### 2.12. Statistical Analysis

Statistical analyses were presented utilizing GraphPad Prism 8.0 software (GraphPad Inc., La Jolla, CA, USA). Data are expressed as the mean ± standard deviation (SD). Comparisons between different groups were performed using Student' s *t*-test or ANOVA followed by Tukey's test. *p* < 0.05 was set as the cutoff criterion.

## 3. Results

### 3.1. Highly Expressed HO-1, Nrf2, MCU, MICU1, and MICU2 in OSCC Tissues

In this study, we determined HO-1, Nrf2, MCU, MICU1, and MICU2 expression in OSCC and normal tissues using immunohistochemistry. Among them, HO-1 and Nrf2 have been confirmed as oncogenes of OSCC [24]. Consistent with previous research, our data confirmed that HO-1 and Nrf2 were highly expressed in OSCC tissues as compared to controls (Figures 1(a) and 1(b)). Nevertheless, the expression of MCU, MICU1, and MICU2 in OSCC remains unclear. Our immunohistochemistry results showed that MCU, MICU1, and MICU2 were all overexpressed in OSCC tissues compared to normal tissues (Figures 1(a) and 1(b)). All of them were mainly expressed in the cytoplasm.

### 3.2. Abnormally Expressed VEGF, TGF-*β*, HIF-1*α*, N-cadherin, and E-cadherin in OSCC

Proteins related to malignant biological behaviors were detected using immunohistochemistry, including VEGF, TGF-*β*, HIF-1*α*, N-cadherin, and E-cadherin. Among them, VEGF, TGF-*β*, HIF-1*α*, and N-cadherin were all overexpressed in OSCC tissues in comparison to normal tissues (Figures 2(a) and 2(b)). E-cadherin was lowly expressed in OSCC tissues compared to normal tissues (Figures 2(a) and 2(b)). These findings indicated that OSCC cells could possess malignant biological behaviors.

### 3.3. Knockdown of MCU or Nrf2 Inhibits Proliferation of OSCC Cells

In view of the high expression of MCU and Nrf2 in OSCC, this study established a stable transfected cell line by spermine treatment and si-MCU transfection in CAL 27 cells. By transfecting sh-Nrf2 in CAL 27 cells, a stable transfected cell line was also built. First, we assessed the influence of different intervention factors on the expression of MCU and Nrf2 in cells by western blot. Our results showed that the control DMSO, Lipofectamine 2000, and GFP-Puro did not change the expression of MCU and Nrf2 (Figures 3(a)–3(c)). Two siRNAs targeting MCU were utilized to transfect CAL 27 cells. Western blot results showed that si-MCU#2 could efficiently silence MCU expression, which was used for the next assays (Figures 3(d) and 3(e)). After transfection with sh-Nrf2#2, Nrf2 expression was distinctly decreased in CAL 27 cells (Figures 3(f)–3(h)). The clone formation assay was utilized to detect the proliferative capacity of cells. The results showed the knockdown of MCU or Nrf2, and the number of CAL 27 cell clones was significantly reduced compared with controls, suggesting that MCU or Nrf2 can enhance the proliferation ability of OSCC cells (Figures 3(i) and 3(j)).

### 3.4. Knockdown of Nrf2 Reverses the Enhancement in Migration Ability Induced by MCU Activation in OSCC Cells

To further explore whether MCU and Nrf2 can affect the migration ability of OSCC cells in vitro, the transwell and scratch experiments were presented to evaluate cell migration ability. Transwell experimental results confirmed that exogenous overexpression of MCU induced by spermine strengthened the migration ability of CAL 27 cells, which was statistically significant (Figures 4(a) and 4(b)). Knockdown of MCU significantly inhibited migration of CAL 27 cells, and sh-Nrf2 also got similar results. Compared with the spermine group, the migration ability of CAL 27 cells was significantly weakened after cotreatment with spermine and sh-Nrf2. Compared with the sh-Nrf2 group, the migration capacity of CAL 27 cells did not significantly change following treatment with spermine and sh-Nrf2, suggesting that MCU could accelerate the migration of OSCC cells, which was regulated by Nrf2. The scratch experiment also confirmed that after overexpression of MCU, migration of CAL 27 cells was distinctly enhanced (Figures 5(a) and 5(b)). The opposite result was observed when silencing MCU or Nrf2. Overexpression of MCU did not change the decrease in cell migration caused by Nrf2 knockdown. However, silencing Nrf2 significantly reduced the enhancement of cell migration caused by MCU overexpression. These findings indicated that silencing Nrf2 could reverse the enhancement in migration ability induced by MCU activation in OSCC cells.

### 3.5. Silencing Nrf2 Decreases the Reinforcement in Mitochondrial Membrane Potential Induced by MCU Activation in OSCC Cells

The level of mitochondrial membrane potential can often reflect whether the function of mitochondria is normal. Therefore, in this experiment, the JC-1 method was used to detect changes in the MMP of each group of cells. As shown in Figures 6(a) and 6(b), the MMP of CAL 27 cells treated with spermine was significantly higher than that of the control group, suggesting that spermine can significantly reduce mitochondrial damage and protect the function of mitochondria. Compared with the control group, when transfected with sh-Nrf2 or si-MCU, the MMP of CAL 27 cells was significantly reduced, suggesting that mitochondrial function was significantly impaired after silencing Nrf2 or MCU. Compared with the spermine treatment group, after treatment of spermine and sh-Nrf2 at the same time, the MMP of the cells was significantly reduced, suggesting that silencing Nrf2 can decrease the protection of spermine to mitochondria. Compared with the sh-Nrf2 group, after cotreatment with spermine and sh-Nrf2, the MMP of the cells was significantly increased, suggesting that spermine can reverse the mitochondrial damage caused by silencing Nrf2. Compared with the control group, the MMP of CAL 27 cells did not change significantly after cotreatment with spermine and sh-Nrf2. These results showed that knockdown of Nrf2 decreased the reinforcement in MMP induced by MCU activation in OSCC cells.

### 3.6. Knockdown of Nrf2 Changes MICU1, MICU2, Vimentin, and N-cadherin Expression Induced by MCU Activation in OSCC Cells

Western blot was presented to detect the expression of HO-1, MCU, MICU1, MICU2, Nrf2, vimentin, N-cadherin, and E-cadherin in CAL 27 cells under different treatments (Figure 7(a)). Compared to controls, HO-1 expression was significantly lower in the sh-Nrf2 transfection group (Figure 7(b)). After overexpressing or silencing MCU, HO-1 expression did not significantly change. Thus, spermine treatment did not change the inhibitory effect of HO-1 expression induced by Nrf2 knockdown (Figure 7(b)). Intriguingly, sh-Nrf2 transfection distinctly decreased MCU expression in CAL 27 cells in comparison to controls (Figure 7(b)). Moreover, spermine did not affect the inhibitory effect of MCU expression induced by sh-Nrf2 treatment, suggesting that MCU expression could be directly mediated by Nrf2. MICU1 and MICU2 expression was distinctly activated in CAL 27 cells treated with spermine, which was suppressed after transfection with si-MCU or sh-Nrf2 (Figure 7(c)). There was no significant difference in MICU1 and MICU2 expression between sh-Nrf2 and sh-Nrf2+spermine groups (Figure 7(c)). However, Nrf2 knockdown significantly reversed the increase in MICU1 and MICU2 expression by spermine (Figure 7(c)), indicating that Nrf2 could promote MICU1 and MICU2 expression via mediating MCU. In Figure 7(d), we found that abnormally expressed MCU did not affect Nrf2 expression in CAL 27 cells. Combining previous findings, we demonstrated that MCU could be a downstream of Nrf2. Compared to controls, vimentin and N-cadherin expression was notably increased in CAL 27 cells treated with spermine, which was decreased following transfection with si-MCU or sh-Nrf2 (Figures 7(d) and 7(e)). Furthermore, silencing Nrf2 prominently reversed the increase in vimentin and N-cadherin expression in CAL 27 cells. Nevertheless, spermine treatment did not change the inhibitory effect of sh-Nrf2 transfection on vimentin and N-cadherin expression (Figures 7(d) and 7(e)). In Figure 7(e), E-cadherin expression was significantly increased in CAL 27 cells under si-MCU or sh-Nrf2 transfection. These results indicated that MCU could be transcriptionally mediated by Nrf2. Furthermore, silencing Nrf2 could alter MICU1, MICU2, vimentin, and N-cadherin expression induced by MCU activation in CAL 27 cells.

### 3.7. Nrf2 Reverses the Increase in MICU1 and MICU2 Expression Induced by MCU Activation in OSCC Cells

In this study, we detected MCU, MICU1, MICU2, and Nrf2 expression in CAL 27 cells under different treatments using immunohistochemistry and immunofluorescence assays. Consistent with western blot results, MCU expression was suppressed after transfection with sh-Nrf2 (Figures 8(a) and 8(b)). Spermine treatment did not change the inhibitory effect of sh-Nrf2. Conversely, Nrf2 knockdown significantly reversed the increase in MCU expression induced by spermine. As shown in Figures 8(c) and 8(d), MICU1 and MICU2 expression was activated after treatment with spermine and was decreased following transfection with si-MCU or sh-Nrf2 in CAL 27 cells. When cotransfected with sh-Nrf2 and spermine, MICU1 and MICU2 expression was distinctly decreased in comparison to that when treated with spermine. However, no significant difference was found between sh-Nrf2+spermine and sh-Nrf2 groups. In Figure 8(e), Nrf2 expression was not significantly affected by MCU overexpression or knockdown in CAL 27 cells. Furthermore, we performed immunofluorescence to detect MCU, MICU1, MICU2, and Nrf2 expression in CAL 27 cells treated with si-MCU or spermine (Figures 9(a)–9(c)). The results showed that MCU (Figure 9(d)), MICU1 (Figure 9(e)), and MICU2 (Figure 9(f)) expression was significantly inhibited by si-MCU, which was distinctly activated by spermine in CAL 27 cells. However, Nrf2 expression was not affected by si-MCU or spermine (Figure 9(g)). These findings revealed that Nrf2 reversed the increase in MICU1 and MICU2 expression induced by MCU activation in OSCC cells.

## 4. Discussion

In line with histopathological examinations, OSCC is featured by squamous differentiation, nuclear polymorphism, and invasive growth [25]. In-depth understanding of the pathogenesis of OSCC and revealing oncogenes and tumor suppressor genes will help improve and supplement the treatment strategies of OSCC, which has important clinical significance. In this study, we found that MCU could participate in the progression of OSCC, which could be regulated by Nrf2. Targeting Nrf2 could simultaneously inhibit MCU and its downstream targets, thereby inhibiting malignant biological behaviors of OSCC cells.

The balance of cell proliferation and cell death is very necessary to maintain the normal growth and development of the body. This kind of balance disorder will cause tumors and other related diseases. Promoting the rapid apoptosis of tumor cells is an effective way to treat tumors. The decrease in mitochondrial membrane potential is often a landmark event in the early stage of apoptosis. In this study, MCU knockdown significantly inhibited the proliferation and induced apoptosis of CAL 27 cells. The deletion of MCU reduces cell proliferation in vivo and in vitro [26]. Local recurrence and metastasis of tumors are important causes of death in OSCC patients. Tumor invasion and metastasis are complex multistep biological processes controlled by various factors. How to effectively inhibit tumor growth and its early metastasis is the key to improving the survival rate of human OSCC patients. Loss of MCU distinctly decreased the migrated capacities of CAL 27 cells. Converse results were observed when MCU was overexpressed. MCU is related to the migration of hepatocellular carcinoma cells [17], breast cancer cells [27], colorectal cancer cells [18], and renal cancer cells [28]. The epithelial-mesenchymal transition (EMT) process was activated by EMT effectors including vimentin, N-cadherin, and E-cadherin in OSCC [29]. Our study found that MCU could speed up the EMT process, thereby inducing migration and invasion of OSCC cells [30].

Nrf2 was activated in OSCC tissues and cells, as in previous studies [31]. Silencing Nrf2 inhibited proliferation and migration and induced apoptosis for OSCC cells. High Nrf2 expression is positively correlated with lymph node metastasis and TNM stage for OSCC patients [24]. Consistently, it has been reported that Nrf2 is involved in the growth and apoptosis of human oral cancer cells [32]. Nrf2, as a transcription factor, could activate the expression of MCU protein. The reinforcement in proliferative and migrative capacities induced by MCU activation was reversed by Nrf2 knockdown. These results suggested that MCU could become a downstream target of Nrf2.

Mitochondrial Ca^2+^ homeostasis is closely related to the occurrence of malignant tumors, including OSCC [33]. The MCU complex plays a critical role in maintaining Ca^2+^ homeostasis. The MICU1-MICU2 heterodimer complex confers Ca^2+^-dependent regulation [34]. MICU1 could prevent mitochondrial calcium overload and mediate tumor growth [35]. Our results showed that MCU could positively regulate the expression of both OSCC cells. Targeting Nrf2 could simultaneously inhibit the expression of MCU, MICU1, and MICU2, thereby maintaining mitochondrial Ca^2+^ homeostasis. Consistently, HO-1 could be regulated by the Nrf2 transcription factor [36]. Targeting the Nrf2/HO-1 axis can delay the growth and metastasis of OSCC [24]. We also found that MCU positively mediated HO-1 expression in OSCC cells, thereby accelerating the progression of OSCC. Furthermore, our data showed that targeting Nrf2 could inhibit EMT of OSCC cells, consistent with previous studies [37]. Knockdown of Nrf2 could reverse the reinforcement in the EMT process induced by MCU activation in OSCC cells.

In conclusion, our research identified that MCU was a novel oncogene for OSCC, which was transcriptionally regulated by Nrf2. MCU accelerated proliferation and migration and inhibited apoptosis for OSCC cells. Thus, MCU could become a novel therapeutic target for OSCC.

## 5. Conclusion

In this study, MCU induced malignant biological behaviors of OSCC cells, which could be regulated by Nrf2. Our findings might provide new molecular targets for targeted therapy of OSCC, as a theoretical and experimental basis for the development of drugs for the prevention and treatment of OSCC.

## Figures and Tables

**Figure 1:** Immunohistochemistry detecting HO-1, Nrf2, MCU, MICU1, and MICU2 expression in OSCC and normal tissues. (a) Representative images of immunohistochemistry results. Bar value = 20 *μ*m. Magnification: 200×. (b) HO-1, Nrf2, MCU, MICU1, and MICU2 expression was quantified according to immunohistochemistry results. ^∗∗∗^*p* < 0.001; ^∗∗∗∗^*p* < 0.0001.

**Figure 2:** Immunohistochemistry detecting VEGF, TGF-*β*, HIF-1*α*, N-cadherin, and E-cadherin expression in OSCC and normal tissues. (a) Representative images of immunohistochemistry results. Bar value = 20 *μ*m. Magnification: 200×. (b) VEGF, TGF-*β*, HIF-1*α*, N-cadherin, and E-cadherin expression was quantified according to immunohistochemistry results. ^∗∗∗^*p* < 0.001; ^∗∗∗∗^*p* < 0.0001.

**Figure 3:** Knockdown of MCU or Nrf2 inhibits the proliferation of OSCC cells. (a–c) MCU expression was detected in CAL 27 cells under different intervention factors using western blot. (d–g) Transfection effects were assessed in CAL 27 cells transfected with si-MCU or sh-Nrf2 by western blot. (h) Representative images of the immunofluorescence assay detecting Nrf2 expression in CAL 27 cells following transfection with sh-Nrf2. Bar value = 100 *μ*m. Magnification: 400×. (i, j) The number of clones for transfected CAL 27 cells. ^∗∗∗^*p* < 0.001; ^∗∗∗∗^*p* < 0.0001; ns: no statistical significance.

**Figure 4:** Transwell results showed that knockdown of Nrf2 could reverse the enhancement in migration ability induced by MCU activation in OSCC cells. (a) Representative images of transwell results. Bar value = 20 *μ*m. Magnification: 200×. (b) The number of migrated cells was counted. ^∗∗∗∗^*p* < 0.0001; ns: no statistical significance.

**Figure 5:** Scratch assay suggested that knockdown of Nrf2 could reverse the enhancement in migration ability induced by MCU activation in OSCC cells. (a) Representative images of the scratch assay. Bar value = 20 *μ*m. Magnification: 200×. (b) The wound distance was measured. ^∗∗^*p* < 0.01; ^∗∗∗^*p* < 0.001; ^∗∗∗∗^*p* < 0.0001; ns: no statistical significance.

**Figure 6:** The effects of Nrf2 and MCU on mitochondrial membrane potential of OSCC cells. (a) Representative images of JC-1 MMP detection results. (b) MMP levels were quantified in CAL 27 cells transfected with spermine, sh-Nrf2, or si-MCU. Magnification: 200×. ^∗∗^*p* < 0.01; ^∗∗∗^*p* < 0.001; ^∗∗∗∗^*p* < 0.0001; ns: no statistical significance.

**Figure 7:** Knockdown of Nrf2 changes MICU1, MICU2, vimentin, and N-cadherin expression induced by MCU activation in OSCC cells. (a) Representative images of western blot results. (b) HO-1 and MCU, (c) MICU1 and MICU2, (d) Nrf2 and vimentin, and (e) N-cadherin and E-cadherin expression was quantified in CAL 27 cells transfected with spermine, sh-Nrf2, or si-MCU. ^∗∗^*p* < 0.01; ^∗∗∗^*p* < 0.001; ^∗∗∗∗^*p* < 0.0001; ns: no statistical significance.

**Figure 8:** Immunohistochemistry assay detecting MCU, MICU1, MICU2, and Nrf2 expression in CAL 27 cells under different treatments. (a) Representative images of immunohistochemistry results. (b) MCU, (c) MICU1, (d) MICU2, and (e) Nrf2 expression was quantified in transfected CAL 27 cells. ^∗∗^*p* < 0.01; ^∗∗∗^*p* < 0.001; ^∗∗∗∗^*p* < 0.0001; ns: no statistical significance.

**Figure 9:** Immunofluorescence assay detecting MCU, MICU1, MICU2, and Nrf2 expression in CAL 27 cells treated with si-MCU or spermine. (a–c) Representative images of immunofluorescence results. (d) MCU, (e) MICU1, (f) MICU2, and (g) Nrf2 expression was quantified in transfected CAL 27 cells. ^∗^*p* < 0.05; ^∗∗^*p* < 0.01; ^∗∗∗^*p* < 0.001; ^∗∗∗∗^*p* < 0.0001.

**Table 1:** Sequences of shRNAs and siRNAs.

Name	Sequences
sh-Nrf2#1	5′-GATCCGCCGGCATTTCACTAAACACAATTCAAGAGATTGTGTTTAGTGAAATGCCGGTTTTTTG-3′
sh-Nrf2#2	5′-GATCCCCGGCCTGCTACTTTAAGCCATTTTCAAGAGAAATGGCTTAAAGTAGCAGGTTTTTTG-3′
si-MCU#1	5′-CAUAAAGGAGCCAAAAAGUCA-3′
si-MCU#2	5′-CGACCUAGAGAAAUACAAUCAGCTC-3′

## Data Availability

The datasets analyzed during the current study are available from the corresponding author on reasonable request.

## Abbreviations

MCU: Mitochondrial calcium uniporter
OSCC: Oral squamous cell carcinoma
Nrf2: Nuclear factor erythroid 2-related factor 2
MICU: Mitochondrial calcium uptake
MMP: Mitochondrial membrane potential
EMT: Epithelial-mesenchymal transition.

## References

[1] Wei M., Wu Y., Liu H., Xie C. (2020). Genipin induces autophagy and suppresses cell growth of oral squamous cell carcinoma via PI3K/AKT/MTOR pathway. *Drug Design, Development and Therapy*.

[2] Gao Z., Zhang Y., Zhou H., Lv J. (2020). Baicalein inhibits the growth of oral squamous cell carcinoma cells by downregulating the expression of transcription factor Sp1. *International Journal of Oncology*.

[3] Bray F., Ferlay J., Soerjomataram I., Siegel R. L., Torre L. A., Jemal A. (2018). Global cancer statistics 2018: GLOBOCAN estimates of incidence and mortality worldwide for 36 cancers in 185 countries. *CA: a Cancer Journal for Clinicians*.

[4] Siegel R. L., Miller K. D., Jemal A. (2019). Cancer statistics, 2019. *CA: a Cancer Journal for Clinicians*.

[5] Chai A. W. Y., Lim K. P., Cheong S. C. (2020). Translational genomics and recent advances in oral squamous cell carcinoma. *Seminars in Cancer Biology*.

[6] Marur S., Forastiere A. A. (2016). Head and neck squamous cell carcinoma: update on epidemiology, diagnosis, and treatment. *Mayo Clinic Proceedings*.

[7] Kain J. J., Birkeland A. C., Udayakumar N. (2020). Surgical margins in oral cavity squamous cell carcinoma: current practices and future directions. *Laryngoscope*.

[8] Chien M. H., Yang W. E., Yang Y. C. (2020). Dual targeting of the p38 MAPK-HO-1 Axis and cIAP1/XIAP by demethoxycurcumin triggers caspase-mediated apoptotic cell death in oral squamous cell carcinoma cells. *Cancers (Basel)*.

[9] Li Y., Liu K., Ke Y. (2019). Risk factors analysis of pathologically confirmed cervical lymph nodes metastasis in oral squamous cell carcinoma patients with clinically negative cervical lymph node: results from a cancer center of Central China. *Journal of Cancer*.

[10] Lalla R. V., Treister N., Sollecito T. (2017). Oral complications at 6 months after radiation therapy for head and neck cancer. *Oral Diseases*.

[11] Peigné L., Godey F., le Gallo M. (2020). One-step nucleic acid amplification for detecting lymph node metastasis of head and neck squamous cell carcinoma. *Oral Oncology*.

[12] Solomon B., Young R. J., Rischin D. (2018). Head and neck squamous cell carcinoma: genomics and emerging biomarkers for immunomodulatory cancer treatments. *Seminars in Cancer Biology*.

[13] Nemani N., Shanmughapriya S., Madesh M. (2018). Molecular regulation of MCU: implications in physiology and disease. *Cell Calcium*.

[14] Vultur A., Gibhardt C. S., Stanisz H., Bogeski I. (2018). The role of the mitochondrial calcium uniporter (MCU) complex in cancer. *Pflügers Archiv*.

[15] Colwill K., Gräslund S. (2011). A roadmap to generate renewable protein binders to the human proteome. *Nature Methods*.

[16] Tosatto A., Sommaggio R., Kummerow C. (2016). The mitochondrial calcium uniporter regulates breast cancer progression via HIF-1*α*. *EMBO Molecular Medicine*.

[17] Ren T., Zhang H., Wang J. (2017). MCU-dependent mitochondrial Ca^2+^ inhibits NAD^+^/SIRT3/SOD2 pathway to promote ROS production and metastasis of HCC cells. *Oncogene*.

[18] Sun Y., Li M., Liu G. (2020). The function of Piezo1 in colon cancer metastasis and its potential regulatory mechanism. *Journal of Cancer Research and Clinical Oncology*.

[19] McMahon M., Lamont D. J., Beattie K. A., Hayes J. D. (2010). Keap1 perceives stress via three sensors for the endogenous signaling molecules nitric oxide, zinc, and alkenals. *Proceedings of the National Academy of Sciences of the United States of America*.

[20] Ohkoshi A., Suzuki T., Ono M., Kobayashi T., Yamamoto M. (2013). Roles of Keap1-Nrf2 system in upper aerodigestive tract carcinogenesis. *Cancer Prevention Research (Philadelphia, Pa.)*.

[21] Chang C. W., Chen Y. S., Tsay Y. G. (2018). ROS-independent ER stress-mediated NRF2 activation promotes Warburg effect to maintain stemness-associated properties of cancer-initiating cells. *Cell Death & Disease*.

[22] Fan H., Paiboonrungruan C., Zhang X. (2017). Nrf2 regulates cellular behaviors and Notch signaling in oral squamous cell carcinoma cells. *Biochemical and Biophysical Research Communications*.

[23] World Medical Association (2013). World Medical Association Declaration of Helsinki: Ethical principles for medical research involving human subjects. *JAMA*.

[24] Liu R., Peng J., Wang H. (2018). Oxysophocarpine retards the growth and metastasis of oral squamous cell carcinoma by targeting the Nrf2/HO-1 axis. *Cellular Physiology and Biochemistry*.

[25] Wu Q. Q., Zhao M., Huang G. Z. (2020). Fibroblast activation protein (FAP) overexpression induces epithelial-mesenchymal transition (EMT) in oral squamous cell carcinoma by down-regulating dipeptidyl peptidase 9 (DPP9). *Oncotargets and Therapy*.

[26] Koval O. M., Nguyen E. K., Santhana V. (2019). Loss of MCU prevents mitochondrial fusion in G1-S phase and blocks cell cycle progression and proliferation. *Science Signaling*.

[27] Tang S., Wang X., Shen Q. (2015). Mitochondrial Ca^2+^ uniporter is critical for store- operated Ca^2+^ entry-dependent breast cancer cell migration. *Biochemical and Biophysical Research Communications*.

[28] Patergnani S., Guzzo S., Mangolini A., Dell’Atti L., Pinton P., Aguiari G. (2020). The induction of AMPK-dependent autophagy leads to P53 degradation and affects cell growth and migration in kidney cancer cells. *Experimental Cell Research*.

[29] Santiago L., Daniels G., Wang D., Deng F. M., Lee P. (2017). Wnt signaling pathway protein LEF1 in cancer, as a biomarker for prognosis and a target for treatment. *American Journal of Cancer Research*.

[30] Dai B. W., Yang Z. M., Deng P. (2019). HOXC10 promotes migration and invasion via the WNT-EMT signaling pathway in oral squamous cell carcinoma. *Journal of Cancer*.

[31] Matsuoka Y., Nakayama H., Yoshida R. (2016). IL-6 controls resistance to radiation by suppressing oxidative stress via the Nrf2-antioxidant pathway in oral squamous cell carcinoma. *British Journal of Cancer*.

[32] Lee Y. M., Auh Q. S., Lee D. W. (2013). Involvement of Nrf2-Mediated Upregulation of Heme Oxygenase-1 in Mollugin- Induced Growth Inhibition and Apoptosis in Human Oral Cancer Cells. *BioMed Research International*.

[33] Cui C., Merritt R., Fu L., Pan Z. (2017). Targeting calcium signaling in cancer therapy. *Acta Pharmaceutica Sinica B*.

[34] Wang C., Jacewicz A., Delgado B. D., Baradaran R., Long S. B. (2020). Structures reveal gatekeeping of the mitochondrial Ca2+ uniporter by MICU1-MICU2. *eLife*.

[35] Marchi S., Corricelli M., Branchini A. (2019). Akt-mediated phosphorylation of MICU1 regulates mitochondrial Ca2+ levels and tumor growth. *The EMBO Journal*.

[36] Piechota-Polanczyk A., Kopacz A., Kloska D. (2018). Simvastatin treatment upregulates HO-1 in patients with abdominal aortic aneurysm but independently of Nrf2. *Oxidative Medicine and Cellular Longevity*.

[37] Feng R., Morine Y., Ikemoto T. (2018). Nrf2 activation drive macrophages polarization and cancer cell epithelial-mesenchymal transition during interaction. *Cell Communication and Signaling: CCS*.

